# Minimal residual disease detected by droplet digital PCR in peripheral blood stem cell grafts has a prognostic impact on high-risk neuroblastoma patients

**DOI:** 10.1016/j.heliyon.2022.e10978

**Published:** 2022-10-08

**Authors:** Nanako Nino, Toshiaki Ishida, Naoko Nakatani, Kyaw San Lin, Kaung Htet Nay Win, Cho Yee Mon, Akihiro Nishimura, Shotaro Inoue, Akihiro Tamura, Nobuyuki Yamamoto, Suguru Uemura, Atsuro Saito, Takeshi Mori, Daiichiro Hasegawa, Yoshiyuki Kosaka, Kandai Nozu, Noriyuki Nishimura

**Affiliations:** a Department of Pediatrics, Kobe University Graduate School of Medicine, Kobe, Japan; b Department of Hematology and Oncology, Kobe Children's Hospital, Kobe, Japan; c Department of Public Health, Kobe University Graduate School of Health Science, Kobe, Japan

**Keywords:** Neuroblastoma (NB), Minimal residual disease (MRD), Peripheral blood stem cell (PBSC), Neuroblastoma-associated mRNAs (NB-mRNAs), Droplet digital PCR (ddPCR)

## Abstract

More than half of high-risk neuroblastoma (NB) patients have experienced relapse due to the activation of chemoresistant minimal residual disease (MRD) even though they are treated by high-dose chemotherapy with autologous peripheral blood stem cell (PBSC) transplantation. Although MRD in high-risk NB patients can be evaluated by quantitative PCR with several sets of neuroblastoma-associated mRNAs (NB-mRNAs), the prognostic significance of MRD in PBSC grafts (PBSC-MRD) is unclear. In the present study, we collected 20 PBSC grafts from 20 high-risk NB patients and evaluated PBSC-MRD detected by droplet digital PCR (ddPCR) with 7NB-mRNAs (CRMP1, DBH, DDC, GAP43, ISL1, PHOX2B, and TH mRNA). PBSC-MRD in 11 relapsed patients was significantly higher than that in 9 non-relapsed patients. Patients with a higher PBSC-MRD had a lower 3-year event-free survival (P = 0.0148). The present study suggests that PBSC-MRD detected by ddPCR with 7NB-mRNAs has a prognostic impact on high-risk NB patients.

## 1 Introduction

Neuroblastoma (NB) is one of the most common solid tumors in children. It originates from neural crest-derived sympathoadrenal progenitors [1, 2, 3] and shows extreme heterogeneity, ranging from spontaneous regression to malignant progression [4, 5]. Approximately half of newly diagnosed NB patients are assigned to a high-risk group and total NB patients account for ∼15% of pediatric cancer-associated deaths. High-risk NB patients are treated by the standard regimen consisting of induction chemotherapy, high-dose chemotherapy with autologous peripheral blood stem cell (PBSC) transplantation, surgery, radiotherapy, and immunotherapy [6, 7]. Although as many as 20% of high-risk NB patients have residual disease that is refractory or progressive [7, 8], the rest of the patients usually achieve remission during induction chemotherapy but potentially have the minimal residual disease (MRD) that causes relapse after completion of the standard regimen [9]. Consequently, more than half of high-risk NB patients still have experienced progression or relapse with a long-term survival rate of around 50% [10]. Patients with relapsed NB have a dismal outcome with less than a 10% rate of long-term survival [11].

To identify MRD in NB patients, a set of neuroblastoma-associated mRNAs (NB-mRNAs) are commonly quantitated in bone marrow (BM), peripheral blood (PB), or PBSC samples due to the lack of recurrent genomic aberrations in NB cells [12, 13]. Several MRD assays quantitating different NB-mRNAs by quantitative PCR (qPCR) or droplet digital PCR (ddPCR) have been shown to possess a significant prognostic value of MRD in BM samples (BM-MRD) for high-risk NB patients [14, 15, 16, 17, 18]. Although we and others have shown the significantly correlated MRD levels between BM and PB samples [17, 18, 19], the prognostic significance of MRD in PB and PBSC samples (PB-MRD and PBSC-MRD) is still unclear.

Because PB has no or fewer detectable tumor cells by immunocytology even when BM is positive in high-risk NB patients, there may be a reduced risk of contamination with tumor cells in PBSC grafts than in BM grafts [20]. PBSC grafts become the first choice for autologous stem cells to restore hemopoiesis after high-dose chemotherapy in the current protocol for high-risk NB patients [7]. However, it remains elusive whether reinfusion of PBSC grafts contaminated with tumor cells can cause relapse and impact the outcome of high-risk NB patients [21]. There are conflicting reports on a prognostic impact of qPCR-based PBSC-MRD monitoring. PBSC-MRD detected by qPCR with B4GALNT1 or TH mRNA was not statistically associated with unfavorable outcomes [22, 23, 24]. In contrast, high PBSC-MRD detected by qPCR with CHGA, DCX, DDC, PHOX2B, or TH mRNA predicted poor outcome [21, 25]. Furthermore, the opposite prognostic impact of qPCR-based PBSC-MRD monitoring was reported for the same cohort. Although PBSC-MRD detected by qPCR with the commonly used adrenergic (ADRN) NB-mRNAs (CHRNA3, DBH, DDC, PHOX2B, or TH mRNA) was not correlated with the outcome, the newly identified mesenchymal (MES) NB-mRNAs (POSTN or PRRX1 mRNA) enabled PBSC-MRD to be significantly associated with poor event-free survival (EFS) and overall survival (OS) [26, 27].

Although we have shown that ddPCR-based MRD monitoring with 7NB-mRNAs (CRMP1, DBH, DDC, GAP43, ISL1, PHOX2B, and TH mRNAs) has a significant prognostic value for BM samples [18], it remains to be determined for PBSC grafts. In the present study, we performed ddPCR-based MRD monitoring in 20 PBSC grafts and evaluated its clinical impact on high-risk NB patients.

## 2 Patients and methods

### 2.1 NB patients and samples

Twenty high-risk NB patients according to the Children's Oncology Group (COG) Neuroblastoma Risk Stratification System [5, 28] or the International Neuroblastoma Risk Group (INRG) Classification System [29] were included in this study. All patients were diagnosed and treated at Kobe Children's Hospital or Kobe University Hospital between June 2011 and January 2018 based on the JN-H-07 [30], JN-H-11 (UMIN000005045), or JN-H-15 (UMIN000016848) protocol of the Japanese Children's Cancer Group (JCCG) Neuroblastoma Committee (JNBSG). All PBSC grafts with written informed consent were harvested after three or four induction cycles when histological tumor content was absent in BM. The present study was conducted in accordance with the guidelines for Clinical Research of Kobe University Graduate School of Medicine with the approval of the Ethics Committee at Kobe University Graduate School of Medicine (No.180278) and Kobe Children's Hospital (No.30-80).

### 2.2 7NB-mRNAs ddPCR assay

7NB-mRNAs ddPCR assay was carried out as described previously [18, 19, 31]. Briefly, total RNA was extracted from PBSC samples using a TRIzol Plus RNA purification kit (Life Technologies, Carlsbad, CA). cDNA was synthesized from 1 μg or 0.5 μg total RNA with a Quantitect reverse transcription kit (Qiagen, Valencia, CA, USA) and stored at −80°C until use. The expression of 7 NB-mRNAs (CRMP1, DBH, DDC, GAP43, ISL1, PHOX2B, and TH) and a reference gene mRNA (HPRT1) was quantitated by a QX200 ddPCR system (Bio-Rad Laboratories, Hercules, CA) according to the digital MIQE (Minimum Information for Publication of Quantitative Digital PCR Experiments) guideline [32, 33]. The level of 7NB-mRNAs (combined signature) was defined as the weighted sum of 7 relative copy numbers (level of each NB-mRNA), in which the reciprocal of 90 percentile in non-NB control PB samples [18] was used for the weighting for each NB-mRNA.

### 2.3 Statistical analysis

The differences in the levels of 7NB-mRNAs between two sample populations were evaluated by the Mann–Whitney U-test. The prognostic value of the levels of 7NB-mRNAs was assessed using the receiver operator characteristic (ROC) analysis. The area under curve (AUC) was interpreted 0.50–0.69 as “low accuracy”, 0.70–0.89 as “moderate accuracy”, and “0.90–1.00” as high accuracy [34]. EFS was defined as the time from the date of diagnosis to the date of relapse or progression. OS was defined as the time from the date of diagnosis to the date of death. EFS and OS were analyzed by the Kaplan–Meier method and log-rank test, and the observation period was censored at 120 months. Reported P values were two-sided and P < 0.05 was considered statistically significant. EZR (version 1.35, www.jichi.ac.jp/saitama-sct/SaitamaHP.files/statmedEN.html; Saitama Medical Center, Jichi Medical University, Saitama, Japan), a modified version of R commander [35], was used for statistical analyses.

## 3 Results

### 3.1 Patient and sample characteristics

Twenty patients included in the present study were all high-risk patients. As summarized in Table 1, these patients had the typical characteristics of high-risk NB: 85% (17/20) were ≧18 months old, 95% (19/20) with INRG stage M, 50% (10/20) with MYCN-amplified tumor, 95% (19/20) with BM metastasis at diagnosis, 80% (16/20) with adrenal gland tumor. All patients were treated according to the JNBSG high-risk NB protocols (JN-H-07, JN-H-11, or JN-H-15) consisting of five cycles of induction chemotherapy and received autologous PBSC grafts as first-line treatment. All PBSC grafts were harvested after three or four cycles of induction chemotherapy when histological tumor content was absent in BM. The median observation time was 47.5 months (range 16–116 months) and a relapse was observed in 55% (11/20) of patients (Figure 1 and Table 1). 3-year EFS and OS were estimated as 45.0% (95% CI: 23.1–64.7%) and 69.3% (95% CI: 44.0–84.9%), respectively (Table 1).

**Table 1:** Patient characteristics.

Age at diagnosis (months)	
Median	32.5
Range	11–75
<18 months	3/20 (15%)
≥18 months	17/20 (85%)

Sex	

Male	15/20 (75%)
Female	5/20 (25%)

INRG stage	

M	19/20 (95%)
L2	1/20 (5%)

MYCN status	

Amplified	10/20 (50%)
Non-amplified	10/20 (50%)

BM metastasis at diagnosis	

Positive	19/20 (95%)
Negative	1/20 (5%)

Primary tumor site	

Adrenal gland	16/20 (80%)
Non-adrenal gland	4/20 (20%)

Observation time (months)	

Median	47.5
Range	16–116

Survival	

3-year EFS	45.0% (95% CI: 23.1–64.7%)
3-year OS	69.3% (95% CI: 44.0–84.9%)

INRG, International Neuroblastoma Risk Group; MYCN, MYCN proto-oncogene, bHLH transcription factor; BM, bone marrow; EFS, event-free survival; OS, overall survival; CI, confidence interval.

**Figure 1:** Clinical course of high-risk NB patients. All patients were subjected to PBSC harvest after three or four cycles of IC and PBSC infusion after HDC. 10 and 1 patients received RA and GD2 for maintenance therapy, respectively. Among 20 patients, 11 patients relapsed and were dead. IC, induction chemotherapy; HDC, high-dose chemotherapy; RT, radiation therapy, RA, 13-cis-retinoic acid; GD2, anti-GD2 antibodies.

### 3.2 PBSC-MRD in high-risk NB patients

To investigate the clinical significance of PBSC-MRD, we first determined the levels of each NB-mRNA (CRMP1, DBH, DDC, GAP43, ISL1, PHOX2B, and TH mRNA) and 7NB-mRNAs by ddPCR in 20 PBSC grafts collected from 20 high-risk NB patients. Consistent with the results obtained from 208 BM and 67 PB samples [18], the levels of each NB-mRNA (Figure 2a) and 7NB-mRNAs (Figure 2b) were detected in 45–75% (9–15/20) and 100% (20/20) of PBSC grafts, respectively, and substantially varied among individual patients.

**Figure 2:** PBSC-MRD in high-risk NB patients. The levels of each NB-mRNA (CRMP1, DBH, DDC, GAP43, ISL1, PHOX2B, and TH mRNA) (a) and 7NB-mRNAs (b) in 20 PBSC grafts were determined by ddPCR.

### 3.3 Association between the level of 7NB-mRNAs in PBSC grafts and relapse of high-risk NB patients

Although the level of 7NB-mRNAs in PBSC grafts was not so high as in BM and PB samples at diagnosis [18], it was significantly higher in PBSC grafts harvested from 11 relapsed patients than in those from 9 non-relapsed patients (Figure 3a). The ROC curve was then plotted for the level of 7NB-mRNAs (Figure 3b). It estimated an AUC of 0.768 with significant accuracy (>0.7), showing that a higher level of 7NB-mRNAs in PBSC grafts predicted relapse of high-risk NB patients.

**Figure 3:** Association between the level of 7NB-mRNAs in PBSC grafts and relapse of high-risk NB patients. (a) The level of 7NB-mRNAs was compared between 9 non-relapsed and 11 relapsed PBSC grafts. (b) The ROC curve was plotted for the level of 7NB-mRNAs in 9 non-relapsed and 11 relapsed PBSC grafts. ROC, the receiver operator characteristic; AUC, the area under curve; TV, threshold value.

### 3.4 Kaplan-Meier curve analysis for high-risk NB patients dichotomized by PBSC-MRD

To clarify the clinical significance of PBSC-MRD, we next performed survival analysis by plotting the Kaplan-Meier curve and estimated 3-year EFS and OS. In the entire cohort of 20 high-risk NB patients, 3-year EFS and OS was 45.0% (95% CI: 23.1–64.7%) and 69.3% (95% CI: 44.0–84.9%), respectively (Table 1). According to the levels of 7NB-mRNAs in PBSC grafts, the entire cohort (n = 20) was dichotomized into MRD-high and MRD-low groups. The cut-off value (7NB-mRNAs = 3.5) was derived from the ROC curve for the level of 7NB-mRNAs (Figure 3b). 3-year EFS (Figure 4a) and OS (Figure 4b) for MRD-high patients (7NB-mRNAs ≧ 3.5, n = 9) vs MRD-low patients (7NB-mRNAs < 3.5, n = 11) was 11.1% (95% CI: 0.6–38.8%) and 55.6% (95% CI: 20.4–80.5%) vs 72.7% (95% CI: 37.1–90.3%) and 81.8% (95% CI: 44.7–95.1%), respectively (p = 0.0148 for EFS and p = 0.18 for OS), suggesting that higher PBSC-MRD was associated with poorer EFS (Figure 4a).

**Figure 4:** Kaplan-Meier curve analysis for high-risk NB patients dichotomized by PBSC-MRD. Kaplan-Meier curve was plotted for EFS (a) and OS (b) of high-risk NB patients with high- and low-PBSC-MRD. EFS, event-free survival; OS, overall survival.

## 4 Discussion

In the present study, we performed ddPCR-based PBSC-MRD monitoring in 20 PBSC grafts with 7NB-mRNAs and revealed that higher PBSC-MRD was significantly associated with poorer EFS in high-risk NB patients. To our knowledge, this is the first study to demonstrate a significant prognostic value of ddPCR-based PBSC-MRD for high-risk NB patients.

A clinical significance of PBSC-MRD remained to be established for high-risk NB patients over the last decades. PBSC-MRD detected by qPCR with B4GALNT1, CHRNA3, DBH, DDC, PHOX2B, or TH mRNA was shown to be not statistically associated with outcome [22, 23, 24, 26], while higher PBSC-MRD detected by qPCR with CHGA, DCX, DDC, PHOX2B, or TH mRNA was reported to be correlated with worse outcome [21, 25]. Compared to qPCR, ddPCR is more sensitive to detect specific nucleic acids and potentially provides more accurate and reproducible quantification of low-level of NB-mRNAs. In the present study, we revealed that higher PBSC-MRD detected by ddPCR with CRMP1, DBH, DDC, GAP43, ISL1, PHOX2B, and TH mRNAs was associated with lower EFS (Figure 4) [18]. Although it is tempting to speculate the superiority of ddPCR for PBSC-MRD monitoring in high-risk NB patients, further validation of ddPCR-based PBSC-MRD monitoring using a larger cohort will be required.

Although NB cells present with very diverse phenotypes, recent studies explored the transcriptomic and epigenetic landscapes of NB cells together with neural crest (NC) cells and identified two super-enhancers (SEs) consisting of dense clusters of enhancers that underlay cell and lineage identity [36, 37, 38]. Based on these SEs, NB cells were classified into two distinct cell states: a neuronal sympathetic ADRN state associated with ADRN NB-mRNAs expression and an undifferentiated and NC-like MES state associated with MES NB-mRNAs expression. These ADRN and MES cells corresponded to the previously described neuroblast (N)-type and substrate-adherent (S)-type cells and had the ability to transdifferentiate or interconvert into each other. In comparison with ADRN cells, MES cells were reported to be more resistant to standard chemotherapeutic drugs such as cisplatin, doxorubicin, and etoposide used to treat NB patients and enriched in post-treatment and recurrent tumors. As MRD was defined as residual tumor cells following local and systemic treatment [39], MES NB-mRNAs were identified and examined for PBSC-MRD detection of high-risk NB patients [27]. Using the same cohort, PBSC-MRD detected by qPCR with MES NB-mRNAs (POSTN or PRRX1 mRNA), but not ADRN NB-mRNAs (CHRNA3, DBH, DDC, PHOX2B, or TH mRNA), was reported to be significantly associated with EFS and OS of high-risk NB patients [26, 27]. In the present study, PBSC-MRD was detected by ddPCR with different ADRN NB-mRNAs (CRMP1, DBH, DDC, GAP43, ISL1, PHOX2B, and TH mRNAs) and was significantly associated with EFS of high-risk NB patients. Further studies using a larger cohort will be required to determine the optimal set of NB-mRNAs (ADRN NB-mRNAs, MES NB-mRNAs, or their combination) for PBSC-MRD detection in high-risk NB patients.

In conclusion, we have revealed that PBSC-MRD detected by ddPCR with 7NB-mRNAs has a significant prognostic value for high-risk NB patients.

## Declarations

### Author contribution statement

Nanako Nino: Performed the experiments, Analyzed and interpreted the data, Contributed reagents, materials, analysis tools, or data, and Wrote the paper.

Toshiaki Ishida; Akihiro Nishimura; Shotaro Inoue; Akihiro Tamura; Nobuyuki Yamamoto; Suguru Uemura; Atsuro Saito; Takeshi Mori: Contributed reagents, materials, analysis tools, or data.

Kyaw San Lin; Kaung Htet Nay Win; Cho Yee Mon: Performed the experiments; Contributed reagents, materials, analysis tools, or data.

Daiichiro Hasegawa; Yoshiyuki Kosaka; Kandai Nozu: Conceived and designed the experiments; Wrote the paper.

Noriyuki Nishimura: Conceived and designed the experiments, Analyzed and interpreted the data, and Wrote the paper.

### Funding statement

Dr. Suguru Uemura and Prof Noriyuki Nishimura were supported by Japan Society for the Promotion of Science [19K17331 & 21K07750].

### Data availability statement

Data included in article/supp. material/referenced in article.

### Declaration of interest’s statement

The authors declare the following conflict of interests: Noriyuki Nishimura received institutional research funding from Sysmex Corporation to Kobe University.

### Additional information

No additional information is available for this paper.
